# Chondroitin sulfatases differentially regulate Wnt signaling in prostate stem cells through effects on SHP2, phospho-ERK1/2, and Dickkopf Wnt signaling pathway inhibitor (DKK3)

**DOI:** 10.18632/oncotarget.22152

**Published:** 2017-10-27

**Authors:** Sumit Bhattacharyya, Leo Feferman, Joanne K. Tobacman

**Affiliations:** ^1^ Department of Medicine, Jesse Brown VA Medical Center, University of Illinois at Chicago, Chicago, IL 60612, USA

**Keywords:** chondroitin sulfate, sulfatase, SHP2, Wnt signaling, phospho-ERK

## Abstract

The chondroitin sulfatases N-acetylgalactosamine-4-sulfatase (ARSB) and galactosamine-N-acetyl-6-sulfatase (GALNS) remove either the 4-sulfate group at the non-reducing end of chondroitin 4-sulfate (C4S) and dermatan sulfate, or the 6-sulfate group of chondroitin 6-sulfate, chondroitin 4,6-disulfate (chondroitin sulfate E), or keratan sulfate. In human prostate cancer tissues, the ARSB activity was reduced and the GALNS activity was increased, compared to normal prostate tissue. In human prostate stem cells, when ARSB was reduced by silencing or GALNS was increased by overexpression, activity of SHP2, the ubiquitous non-receptor tyrosine phosphatase, declined, attributable to increased binding of SHP2 with C4S. This led to increases in phospho-ERK1/2, Myc/Max nuclear DNA binding, DNA methyltransferase (DNMT) activity and expression, and methylation of the Dickkopf Wnt signaling pathway inhibitor (DKK)3 promoter and to reduced DKK3 expression. Since DKK3 negatively regulates Wnt/β-catenin signaling, silencing of ARSB or overexpression of GALNS disinhibited (increased) Wnt/β-catenin signaling. These findings indicate that the chondroitin sulfatases can exert profound effects on Wnt-mediated processes, due to epigenetic effects that modulate Wnt signaling.

## INTRODUCTION

The chondroitin sulfatases, ARSB (Arylsulfatase B; N-acetylgalactosamine-4-sulfatase) and GALNS [galactosamine-(N-acetyl)-6-sulfatase; N-acetylgalactosamine-6-sulfatase; galactose-6-sulfate sulfatase] remove either the 4-sulfate or 6-sulfate group from the non-reducing end of N-acetylgalactosamine sulfate residues. Genetic mutations of these enzymes lead to the lysosomal storage disorders Mucopolysaccharidosis VI (Maroteaux-Lamy-Disease), in which there is genetic mutation of ARSB, or Mucopolysaccharidosis IVA (Morquio A), in which there is genetic mutation of GALNS. These innate disorders are characterized by the widespread accumulation of chondroitin sulfates and other sulfated glycosaminoglycans, since hydrolysis of the sulfate ester at the non-reducing end is required for sulfated GAG degradation [1–6].

In this report, we extend our previous findings about a role for ARSB deficiency in prostate cancer [7, 8]. The experiments in this report show how acquired changes in expression of the chondroitin sulfatases ARSB and GALNS contribute to activation of Wnt/β-catenin signaling by reducing the expression of the Dickkopf Wnt signaling inhibitor DKK3. In other reports, Dickkopf has been identified as a negative regulator of Wnt signaling, possibly due to its interaction with LDL-receptor related protein (LRP) 5/6 to block Wnt binding with its receptor complex at the cell membrane [9–11].

In the experiments presented in this report, the increase in chondroitin 4-sulfate (C4S), which results from decline in ARSB, leads to increased methylation of the DKK3 promoter and reduced DKK3 expression. Also, when GALNS is overexpressed, there is increased methylation of the DKK3 promoter and decline in DKK3. The signaling pathway to inhibition of DKK3 expression by the chondroitin sulfatases proceeds by inhibition of the ubiquitous, non-receptor tyrosine phosphatase SHP2 (PTPN11), which is attributed to increased binding of SHP2 with C4S when ARSB is reduced or GALNS is increased. Previously, SHP2 was shown to co-immunoprecipitate with C4S, and more SHP2 co-immunoprecipitated when ARSB was silenced and C4S was increased [12]. The mechanism by which the SHP2 inhibitor, phenylhydrazonopyrazolone sulfonate (PHPS1), inhibits SHP2 was previously determined to be by mimicry of its sulfonyl group with a phospho-tyrosine binding site of SHP2 [13], and we suggest that the 4-sulfate group of N-acetylgalactosamine 4-sulfate at the non-reducing end of C4S may provide a similar binding site for SHP2.

The sulfation of C4S has been shown to be of great importance in fundamental biological reactivity, including in adhesion of malarial parasites to vascular endothelium and placenta [14, 15] and in neuronal regeneration following injury [16, 17]. In previous reports, other mechanisms by which decline in ARSB may contribute to development of malignancy through transcriptional effects were presented [7, 12, 18-21]. Reduced binding of galectin-3 to the more highly sulfated C4S present when ARSB was reduced was associated with transcriptional events mediated by AP (Activator Protein)-1 and Sp (Specificity protein)1, leading to increased mRNA expression of HIF-1α, versican, Wnt9A, and CSPG4 [7, 12, 19, 20]. Also, increased binding of SHP2 to C4S was associated with increased expression of transmembrane glycoprotein NMB (GPNMB) in hepatic cells [18] and of matrix-metalloproteinase (MMP)-9 in melanomas [12], due to sustained activation of phospho-38 MAPK (mitogen-activated protein kinase) and of phospho-ERK (Extracellular-signal regulated kinase)1/2). In other experiments, increased binding of bone morphogenetic protein (BMP)-4 to the more highly sulfated C4S present when ARSB was silenced modified Smad signaling and reduced the expression of the chondroitin 4-sulfotransferase CHST11 [21].

Decline in ARSB activity was demonstrated in human prostate cancer tissues and in prostate cancer tissue microarrays [7, 8]. Less intense ARSB immunochemical staining was associated with more aggressive prostate cancers, with higher Gleason scores, and with earlier recurrence [8]. The increased expression of the extracellular matrix proteoglycan versican, which has epidermal growth factor (EGF)-like domains, was associated with increased BrdU (5-bromo-2'-deoxyuridine) incorporation, following exposure to exogenous EGF in prostate epithelial cells [7]. This suggested that changes in ARSB and in C4S might contribute to increased proliferation in prostate cancer. Other investigators have also identified increased versican and increased chondroitin sulfate in association with prostate cancer progression or more aggressive disease [22–24]. In other studies, decreased ARSB activity was linked to enhanced aerobic glycolysis, the Warburg effect, due to impaired oxidative metabolism, increased lactate production, and mitochondrial abnormalities in human hepatic cells and in hepatic tissue of ARSB-null mice [25].

With this background, further investigation of the impact of changes in chondroitin sulfatases and in chondroitin sulfate in prostate stem cells was initiated. Initial studies focused on how changes in activity of the chondroitin sulfatases modified known targets of Wnt signaling, including nuclear β-catenin, nuclear DNA-bound TCF/LEF (T-cell factor/Lymphoid enhancing factor), and mRNA expression of c-Myc and GATA-3 [26, 27]. Other preliminary experiments had shown epigenetic effects of the chondroitin sulfatases, with increases in DNA methyltransferase activity and DNA methyltransferase mRNA expression. The experiments presented in this report were performed to identify a signaling pathway involving DNA methylation by which the chondroitin sulfatases impacted on Wnt/β-catenin signaling. Since decline in expression of the Dickkopf Wnt signaling pathway inhibitor (DKK3) increases Wnt/β-catenin signaling [9–11], investigation focused on the epigenetic regulation of DKK3 expression.

## RESULTS

### ARSB and GALNS activity and expression in prostate stem cells and prostate tissues

In human prostate stem cells, ARSB activity decreased to ∼11.5% of the control level 24 h after silencing of ARSB mRNA expression by specific siRNA. ARSB activity increased to ∼235% of the control level 24 h post-transfection of the ARSB plasmid in the pCMV6-XL4 vector (Figure 1A). GALNS activity was not changed significantly from the baseline level after either ARSB silencing or overexpression. GALNS activity declined to ∼11.2% of the control baseline level 24 h post-silencing of GALNS mRNA expression by specific siRNA (Figure 1B). GALNS activity increased to ∼157% of the control baseline level 24 h post transfection with the GALNS plasmid. Neither GALNS silencing nor overexpression had any impact on baseline ARSB activity, reflecting the specificity of silencing and overexpression.

**Figure 1:** ARSB and GALNS in human prostate stem cells and prostate tissue **(A)** ARSB activity was measured in prostate stem cells using the exogenous substrate 4-methylumbelliferyl sulfate. ARSB activity was significantly reduced by ARSB knockdown by specific siRNA and increased by ARSB overexpression using ARSB plasmid in a pCMV6-XL4 vector in the prostate stem cells (p<0.001, n=3). GALNS silencing or overexpression did not affect the ARSB activity. **(B)** GALNS activity was measured using the exogenous substrate 4-methylumbelliferyl-β-D-galactoside-6-sulfateNH_4_. GALNS activity was significantly reduced by GALNS siRNA and increased by GALNS overexpression using GALNS plasmid in a pCMV6-XL4 vector (p<0.001, n=3). ARSB silencing or overexpression did not affect the GALNS activity. **(C)** In malignant prostate tissue, the ARSB activity was significantly lower than in the normal human prostate tissue (p<0.0001, n=6, unpaired t-test, two-tailed). **(D)** In contrast, the GALNS activity was significantly higher in the malignant tissue (p<0.0001, n=6, unpaired t-test, two-tailed). [ARSB = arylsulfatase B = N-acetylgalactosamine-4-sulfatase; GALNS = galactosamine-(N-acetyl)-6-sulfatase; N-acetylgalactosamine-6-sulfatase; galactose-6-sulfate sulfatase; OE = overexpression; si = siRNA].

ARSB and GALNS activity and expression were assessed in normal and malignant human prostate tissues. ARSB activity was significantly lower in the malignant tissue (70.4 ± 4.0 vs. 129.9 ± 12.8 nmol/mg protein/h; p<0.0001 unpaired t-test, two-tailed; n=6) (Figure 1C). In contrast, the GALNS activity was significantly higher in malignant prostate tissue than in the normal tissue (8.1 ± 0.4 vs. 6.4 ± 0.4 nmol/mg protein/h; p<0.0001, unpaired t-test; two-tailed; n=6) (Figure 1D).

### Total sulfated glycosaminoglycan and chondroitin sulfate measurements in prostate stem cells and prostate tissues

Both ARSB and GALNS silencing significantly increased the total sulfated glycosaminoglycan (GAG) content of the prostate stem cells (p<0.001) (Figure 2A), which was measured by the Blyscan™ assay. ARSB silencing induced a ∼74% increase of chondroitin 4-sulfate (C4S) above the baseline level (Figure 2B), whereas chondroitin 6-sulfate (C6S) remained unchanged (Figure 2C). GALNS silencing stimulated a ∼97% increase in C6S, but C4S remained unchanged. The C4S/C6S ratio increased from 1.58 ± 0.07 to 2.57 ± 0.32 after ARSB silencing, and decreased to 0.82 ± 0.08 after GALNS silencing (Figure 2D). The C4S and the C6S were measured by the Blyscan™ assay, following immunoprecipitation of the cell lysate by the C4S or C6S antibody, respectively. The increases in the chondroitin sulfates following silencing of the chondroitin sulfatases are consistent with the critical role of the chondroitin sulfatases in the degradation of the chondroitin sulfates.

**Figure 2:** Total sulfated GAGs, C4S, C6S, and C4S/C6S ratio in human prostate stem cells and prostate tissue **(A)** Total sulfated glycosaminoglycans (GAGs) were measured using the Blyscan™ assay which detects sulfated GAGs by binding to 1,9-dimethylmethylene blue. In the prostate stem cells, total sulfated glycosaminoglycans (GAGs) were increased following silencing of ARSB or of GALNS (p<0.001, n=3). In contrast, overexpression of ARSB or of GALNS decreased the total sulfated GAGs (p<0.001, n=3). **(B)** Chondroitin-4-sulfate (C4S) was measured by the Blyscan™ assay, following immunoprecipitation by antibody specific for C4S. C4S was significantly increased following ARSB silencing and reduced when ARSB was overexpressed (p<0.001, n=3). Changes in GALNS expression did not affect the level of C4S. **(C)** Chondroitin 6-sulfate was detected by the Blyscan™ assay, following immunoprecipitation with an antibody specific for C6S. When GALNS was silenced, chondroitin 6-sulfate (C6S) increased significantly, and declined when GALNS was overexpressed (p<0.001, n=3). Changes in ARSB expression did not affect the C6S level. **(D)** The C4S/C6S ratio was calculated and shown to be increased when ARSB was silenced or GALNS was overexpressed (p<0.001, n=3). The ratio was reduced when ARSB was overexpressed or GALNS was silenced. **(E)** In the human prostate tissues, C6S and C4S were measured by the Blyscan™ assay. C4S was increased and C6S was reduced in the malignant tissue (p<0.001, n=6; unpaired t-test, two-tailed), consistent with decrease in ARSB activity and increase in GALNS activity. Overall, total sulfated GAGs were significantly increased in the malignant tissue, compared to the normal tissue (p<0.01, n=6). **(F)** The C4S/C6S ratio was calculated and was increased in the malignant tissue, compared to the normal tissue (p<0.001, n=6; unpaired t-test, two-tailed). [ARSB=arylsulfatase B=N-acetylgalactosamine-4-sulfatase; C4S=chondroitin 4-sulfate; C6S=chondroitin 6-sulfate; GALNS=galactosamine-(N-acetyl)-6-sulfatase; N-acetylgalactosamine-6-sulfatase; galactose-6-sulfate sulfatase; GAG=glycosaminoglycan; OE=overexpressed; si=siRNA].

In contrast to the effects of silencing, both ARSB and GALNS overexpression significantly reduced the total sulfated GAG content of the prostate stem cells (p<0.001) (Figure 2A). ARSB overexpression reduced the C4S content (Figure 2B), and GALNS overexpression reduced the C6S content (Figure 2C). C4S was unaffected by GALNS silencing or overexpression, and C6S was unaffected by ARSB silencing or overexpression. The C4S/C6S ratio decreased from 1.58 ± 0.07 to 0.42 ± 0.004 after ARSB overexpression and increased to 5.23 ± 0.29 after GALNS overexpression (Figure 2D).

In the malignant prostate tissue, total sulfated GAG and C4S levels were significantly higher, and C6S was significantly lower (p<0.001) than in control prostate tissue (Figure 2E). The C4S/C6S ratio was nearly three times higher in the malignant prostate tissue than in the normal tissue (Figure 2F).

### ARSB silencing and GALNS overexpression lead to increased Wnt/β-catenin signaling

Effects of changes in expression of the chondroitin sulfatases on targets of β-catenin/Wnt signaling were addressed in the prostate stem cells. Both ARSB silencing and GALNS overexpression increased the nuclear concentration of β-catenin (p<0.001, n=3) (Figure 3A). In contrast, ARSB overexpression and GALNS knockdown reduced the nuclear β-catenin. In the malignant prostate tissues, nuclear β-catenin was greater than in the normal tissue (p=0.015, unpaired t-test, two-tailed, n=6) (Figure 3B). Nuclear DNA-bound TCF/LEF, which acts with β-catenin to modulate the expression of Wnt target genes, was increased following ARSB silencing or GALNS overexpression in the prostate stem cells (p<0.001, n=3) (Figure 3C). Inversely, ARSB overexpression and GALNS silencing decreased the nuclear-bound TCF/LEF (Figure 3C).

**Figure 3:** Effects of ARSB and GALNS on Wnt/ß-catenin signaling **(A)** Nuclear β-catenin was measured by ELISA in nuclear extracts of the prostate stem cells following ARSB and GALNS silencing and overexpression. Nuclear ß-catenin increased significantly following ARSB silencing or GALNS overexpression (p<0.001, n=3). Inversely, GALNS silencing or ARSB overexpression reduced the nuclear ß-catenin (p<0.001, n=3). **(B)** Nuclear ß-catenin was measured in nuclear extracts from normal and malignant human prostate tissue. Nuclear ß-catenin was significantly increased in the malignant tissue (p<0.01, unpaired t-test, two-tailed, n=6). **(C)** Nuclear DNA-bound TCF/LEF was determined by a transcription factor reporter assay in the prostate stem cells. A biotin-labeled TCF/LEF DNA binding sequence probe which detected TCF/LEF bound to DNA was mixed with nuclear extracts to form TCF/LEF-DNA complexes. A filter plate was used to retain the bound DNA probe and remove free probe. The bound prelabeled DNA probe was eluted from the filter and collected for quantitative determination. The bound TCF/LEF increased following either ARSB silencing or GALNS overexpression (p<0.001, n=3). In contrast, ARSB overexpression and GALNS silencing inhibited the increase (p<0.001, n=3). **(D)** Further demonstration of the impact of the chondroitin sulfatases was shown by effects on the mRNA expression of Wnt/ß-catenin dependent genes. QPCR showed increased expression of c-Myc and GATA-3 following ARSB silencing or GALNS overexpression. In contrast, overexpression of ARSB or silencing of GALNS reduced the mRNA expression of c-Myc and GATA-3 (p<0.001, n=6). [ARSB=arylsulfatase B=N-acetylgalactosamine-4-sulfatase; C4S=chondroitin 4-sulfate; C6S=chondroitin 6-sulfate; GALNS=galactosamine-(N-acetyl)-6-sulfatase; N-acetylgalactosamine-6-sulfatase; galactose-6-sulfate sulfatase; GAG=glycosaminoglycan; OE=overexpressed; si=siRNA; TCF/LEF=T-cell factor/lymphoid enhancer-binding factor].

ARSB silencing and GALNS overexpression increased the mRNA expression of Wnt/β-catenin target genes, including c-Myc and GATA-3 (p<0.001, n=6) (Figure 3D). Inversely, ARSB overexpression and GALNS silencing inhibited the gene expression (p<0.001, n=6) (Figure 3D).

### Effect of chondroitin sulfatases on targets of Wnt/β-catenin signaling is dependent on DNA methylation

Treatment of the prostate stem cells with the hypomethylating agent 5-azacytidine nullified the stimulatory effect of ARSB silencing or GALNS overexpression on the increases in nuclear β-catenin (Figure 4A), nuclear DNA-bound TCF/LEF (Figure 4B), and c-Myc and GATA-3 gene expression (Figure 4C). These findings are consistent with an underlying epigenetic mechanism leading to the activation of the Wnt signaling pathway following changes in chondroitin sulfates due to decline in ARSB or increase in GALNS.

**Figure 4:** Inhibition of chondroitin sulfatase-induced changes in Wnt/ß-catenin signaling by inhibition of DNA methylation **(A)** When the prostate stem cells were treated with the DNA hypomethylating agent 5-azacytidine (10 μM x 24 h), the ARSB silencing- or GALNS overexpression- induced increases in nuclear β-catenin were inhibited (p<0.001, n=3). This indicated that a transcriptional mechanism was required for the effects of ARSB siRNA and GALNS overexpression on nuclear ß-catenin. **(B)** Similarly, the effects of ARSB silencing or GALNS overexpression on TCF/LEF binding to nuclear DNA were inhibited by treatment with the DNA hypomethylating agent, 5-azacytidine, (p<0.001, n=3). This indicated that a transcriptional mechanism was required for the activation of Wnt/β-catenin signaling, as manifested by effects of ARSB siRNA and GALNS overexpression on TCF/LEF nuclear-DNA binding. **(C)** QPCR was performed using standard quantitative methods and established primers. The increased mRNA expression of c-Myc and of GATA-3 following either ARSB silencing or GALNS overexpression was inhibited by 5-azacytidine (p<0.001, n=6). These effects are consistent with dependence on DNA methylation for the observed increases in manifestations of Wnt/ß-catenin signaling following changes in activity of chondroitin sulfatases ARSB and GALNS. **(D)** Treatment with JW67 (4 mg/ml x 24 h), an inhibitor of the Wnt/ß-catenin signaling pathway, also blocked the ARSB silencing-induced increases in mRNA expression of c-Myc and GATA-3 (p<0.001, n=6). This finding indicates that the increased activation of Wnt/β-catenin signaling was also required to increase the expression of these Wnt target genes. **(E)** The effect of GALNS overexpression on mRNA expression of c-Myc and GATA-3 was also inhibited by JW67 (p<0.001, n=6). This finding indicated that the effects of ARSB silencing and GALNS overexpression on Wnt target genes were both mediated by activation of Wnt/β-catenin signaling. [ARSB=arylsulfatase B=N-acetylgalactosamine-4-sulfatase; 5-AZA=5-azacytidine; GALNS=galactosamine-(N-acetyl)-6-sulfatase; N-acetylgalactosamine-6-sulfatase; galactose-6-sulfate sulfatase; OE=overexpression; si=siRNA; TCF/LEF=T-cell factor/lymphoid enhancer-binding factor].

Effects on the ARSB- and GALNS-mediated changes in the mRNA expression of c-Myc and on GATA-3 were inhibited by both 5-azacytidine (Figure 4C) and JW67 (Figure 4D, 4E), an inhibitor of Wnt/β-catenin pathway activation.

### Chondroitin sulfatases activate Wnt signaling by decreasing Dickkopf (DKK)3 expression

Since activation of Wnt signaling follows the inhibition of DKK3 (Dickkopf inhibitor of Wnt signaling) [9–11], the effects of the chondroitin sulfatases on DKK3 expression were investigated in the prostate stem cells. ARSB silencing and GALNS overexpression inhibited the mRNA expression of DKK3 in the prostate stem cells (Figure 5A). Inversely, ARSB overexpression and GALNS silencing induced the expression of DKK3 mRNA (Figure 5A). Treatment with 5-azacytidine reversed the inhibitory effects of ARSB silencing and GALNS overexpression on DKK3 expression (Figure 5B), indicating that DNA methylation was required for this effect. In contrast to the inhibitory effects of JW67 on the mRNA expression of c-Myc and GATA-3, JW67 did not block the effects of ARSB silencing (Figure 5C) or GALNS overexpression (Figure 5D) on inhibition of DKK3 expression. This indicated that Wnt/β-catenin signaling was not implicated in the impact of the chondroitin sulfatases on DKK3 expression, and was consistent with an epigenetic mechanism regulating the DKK3 expression in the prostate stem cells following changes in the chondroitin sulfatases.

**Figure 5:** Dickkopf inhibitor of Wnt signaling pathway (DKK3) expression is inhibited by ARSB knockdown or GALNS overexpression **(A)** In contrast to the increased expression of c-Myc and GATA-3 when ARSB was silenced or GALNS overexpressed, the mRNA expression of DKK3, an inhibitor of Wnt signaling, was reduced by ARSB silencing or by GALNS overexpression (p<0.001, n=6). Inversely, GALNS silencing and ARSB overexpression increased the DKK3 mRNA (p<0.001, n=6). **(B)** The declines in mRNA expression of DKK3 induced by ARSB silencing or GALNS overexpression were reversed by treatment with 5-azacytidine (10 μM x 24h) (p<0.001, n=6), consistent with dependence on DNA methylation. **(C)** In contrast to the impact of JW67 on mRNA expression of c-Myc and GATA-3, inhibition of the Wnt/ß-catenin signaling pathway by JW67 (4 mg/ml x 24 h) had no impact on the mRNA expression of DKK3 following ARSB silencing (p<0.001, n=6). This indicated that the effect of the chondroitin sulfatases on DKK3 expression was independent of activation of the Wnt/ß-catenin signaling pathway. **(D)** JW67 had no impact on mRNA expression of DKK3 following GALNS overexpression (p<0.001, n=6). **(E)** In the malignant prostate tissue, the DKK3 mRNA was significantly reduced, compared to the level in the normal prostate tissue (p<0.0001, unpaired t-test, two tailed; n=6). **(F)** The DKK3 secreted into the spent media of the prostate stem cells was determined by ELISA. Levels were significantly reduced by either ARSB silencing or GALNS overexpression, and increased when ARSB was overexpressed or GALNS was silenced (p<0.001, n=3). [ARSB=arylsulfatase B=N-acetylgalactosamine-4-sulfatase; 5-AZA=5-azacytidine; DKK=Dickkopf inhibitor of Wnt signaling pathway; GALNS=galactosamine-(N-acetyl)-6-sulfatase; N-acetylgalactosamine-6-sulfatase; galactose-6-sulfate sulfatase; OE=overexpression; si=siRNA].

Consistent with activation of the Wnt signaling pathway in malignancy, DKK3 mRNA was reduced in the malignant prostate tissue, compared to the normal prostate tissue (p<0.0001, unpaired t-test, two-tailed, n=6) (Figure 5E). Both ARSB silencing and GALNS overexpression reduced the protein content of DKK3 in the spent media of the prostate stem cells (p<0.001) (Figure 5F). Inversely, ARSB overexpression and GALNS silencing increased the level of DKK3 protein in the spent media (Figure 5F).

### Determination of DKK3 promoter methylation by methylation-specific QPCR

The epigenetic mechanism by which decline in ARSB or increase in GALNS reduced the expression of DKK3 was investigated. The impact of ARSB and GALNS on methylation of the DKK3 promoter was investigated by methylation-specific QPCR using primers specific for the methylated and unmethylated DKK3 promoter. ARSB silencing and GALNS overexpression increased the DKK3 promoter methylation, in contrast to ARSB overexpression and GALNS silencing which reduced the methylation (Figure 6A). Representative DNA gels demonstrated increased band intensity of the DKK3 promoter following ARSB silencing and GALNS overexpression (Figure 6B). Methylation of the DKK3 promoter in malignant prostate tissue was also significantly increased, compared to the normal tissue (p<0.0001, unpaired t-test, two tailed; n=6) (Figure 6C).

**Figure 6:** DKK3 promoter methylation is increased by ARSB silencing or GALNS overexpression **(A)** Whole genomic DNA from prostate stem cells in which ARSB and GALNS had been silenced or overexpressed and from control samples was obtained and fractionated. Methylated DNA was isolated by binding to the methyl-CpG binding domain of human MBD2 protein, which was coupled to paramagnetic Dynabeads^R^ M-280 Streptavidin via a biotin linker. The methylated fragments were then eluted and subjected to QPCR with specific primers to the DKK3 promoter. DKK3 promoter methylation was increased when ARSB was silenced or GALNS overexpressed (p<0.001, n=6), and reduced when GALNS was silenced or ARSB overexpressed (p<0.001, n=6). **(B)** By methylation specific PCR using primers specific for both the methylated and unmethylated DKK3 promoter, the expression of the methylated DKK3 promoter was demonstrated on a 2% agarose gel. Band density was increased following GALNS overexpression and ARSB silencing (p<0.001, n=3). **(C)** Genomic DNA was isolated from normal and malignant prostate tissue and was fractionated. The methylated dsDNA was isolated by binding to MBD2 which was coupled to Dynabeads, as above. QPCR was performed to quantify the DKK3 promoter methylation. In the malignant prostate tissue, DKK3 promoter methylation was increased (p<0.0001, n=6; unpaired t-test, two-tailed), thereby inhibiting DKK3 expression and permitting increased Wnt signaling. [ARSB=arylsulfatase B=N-acetylgalactosamine-4-sulfatase; DKK=Dickkopf inhibitor of Wnt signaling pathway; GALNS=galactosamine-(N-acetyl)-6-sulfatase; N-acetylgalactosamine-6-sulfatase; galactose-6-sulfate sulfatase; OE=overexpression; si=siRNA].

### Chondroitin sulfatases affect activity and expression of DNA methyltransferases (DNMTs)

To address the mechanism whereby changes in chondroitin sulfatases could modify DKK3 promoter methylation, the impact of ARSB and GALNS on DNA Methyltransferase (DNMT) expression and activity in the prostate stem cells was determined. The mRNA expression of DNMT 1, 3a, and 3b was determined in the prostate stem cells following changes in chondroitin sulfatases by silencing and overexpression of ARSB and GALNS. DNMT 1 and 3a were significantly increased by ARSB silencing and GALNS overexpression, and inversely affected by ARSB overexpression and GALNS knockdown (p<0.001) (Figure 7A).

**Figure 7:** Chondroitin sulfatases modify DNMT expression and activity **(A)** DNMT 1, DNMT 3a, and DNMT 3b mRNA expression was determined by QPCR using established primers. ARSB silencing and GALNS overexpression increased expression of DNMT1 and DNMT3a, and expression of DNMT3b was unaffected. Inversely, GALNS silencing and ARSB overexpression reduced expression of DNMT1 and DNMT3a (p<0.001, n=6). **(B)** DNMT activity was determined in nuclear extracts from control and treated prostate stem cells by the EpiQuik™ DNA Methyltransferase (DNMT) Activity/Inhibition Assay Kit. A unique cytosine-rich DNA substrate was coated onto wells, and DNMT enzymes in the samples transferred a methyl group to the cytosines from exogenous Adomet. The methylated DNA was recognized by an anti-5-methylcytosine antibody. DNMT activity was significantly increased by either ARSB silencing or GALNS overexpression in the prostate stem cells (p<0.001, n=3). Inversely, GALNS silencing and ARSB overexpression inhibited the DNMT activity. **(C)** When the cells were treated with the ERK activation inhibitor peptide I (10 μM x 24 h), the impact of ARSB silencing or of GALNS overexpression on DNMT activity was blocked (p<0.001, n=3). This result indicates a requirement for ERK activation for the DNMT activity. [ARSB=arylsulfatase B=N-acetylgalactosamine-4-sulfatase; DKK=Dickkopf Wnt inhibitory factor 1; DNMT=DNA methyltransferase; ERK=extracellular-signal regulated kinase; GALNS=galactosamine-(N-acetyl)-6-sulfatase; N-acetylgalactosamine-6-sulfatase; galactose-6-sulfate sulfatase; OE=overexpression; si=siRNA].

The DNMT activity was stimulated 79% by ARSB silencing and 66% by GALNS overexpression. Inversely, ARSB overexpression and GALNS silencing reduced the DNMT activity by 42% and 46%, compared to controls (p<0.001) (Figure 7B).

Since the impact of decline in ARSB was mediated by increased phospho-ERK1/2 in other experiments [12], the impact of ERK inhibition on the ARSB-induced increase in DNMT activity was addressed in the prostate stem cells. Treatment with the ERK activation inhibitor peptide I blocked the increase in DNMT activity induced by ARSB silencing and by GALNS overexpression (Figure 7C).

### Impact of chondroitin sulfatases on phospho-ERK1/2 activity is mediated by SHP2

Further assessment of the impact of the chondroitin sulfatases on phospho-ERK1/2 was performed. In the prostate stem cells, phospho-ERK1/2 was markedly increased by silencing ARSB or by the overexpression of GALNS (Figure 8A). The ERK activity inhibitor peptide I was effective in reversing the effect of GALNS OE and ARSB silencing. In the malignant prostate tissue, the phospho-ERK1/2 was significantly increased, compared to the normal prostate tissue (p<0.001, unpaired t-test, two-tailed, n=6) (Figure 8B).

**Figure 8:** Chondroitin sulfatases modify ERK1/2 activity by effects on SHP2 **(A)** Phospho-ERK1/2 was determined by sandwich ELISA, in which total ERK1/2 was first captured in the wells of an ELISA plate. A second antibody was used to detect phospho-ERK1/2. In the prostate stem cells, GALNS overexpression and ARSB silencing increased the phospho-ERK1/2 (p<0.001, n=3). In contrast GALNS silencing and ARSB OE reduced the phospho-ERK1/2 (p<0.001, n=3). The ERK activity inhibitor peptide I was effective in reversing the effect of the GALNS OE and ARSB silencing. **(B)** In human prostate tissue, phospho-ERK1/2 was significantly increased in the malignant tissue, compared to normal (p<0.001, n=6; unpaired t-test, two-tailed). **(C)** Decline in SHP2 activity, due to transfection with a dominant negative SHP2 DNA construct, led to significant increase in phospho-ERK1/2 in the prostate stem cells (p<0.001, n=3). In contrast, the constitutively active SHP2 construct reduced the phospho-ERK1/2 (p<0.001, n=3). **(D)** SHP2 activity was determined by measurement of phosphate released from a synthetic phosphopeptide, following isolation of SHP2 by anti-SHP2 antibody conjugated to agarose beads. ARSB silencing and GALNS overexpression reduced the SHP2 activity in the prostate stem cells (p<0.001, n=3). In contrast, GALNS silencing and ARSB overexpression increased the SHP2 activity (p<0.001, n=3). These effects are attributed to increased binding of SHP2 to C4S when ARSB was silenced or GALNS was overexpressed. **(E)** In the prostate stem cells, ARSB silencing significantly reduced the SHP2 activity. The dominant negative (DN) SHP2 DNA construct further reduced the SHP2 activity (p<0.001, n=3). The effect of ARSB silencing was inhibited by the constitutively active (CA) SHP2 DNA construct (p<0.001, n=3). **(F)** In the malignant human prostate tissue, the SHP2 activity was reduced ∼50% (p<0.001, n=6; unpaired t-test, two-tailed), attributable to the previously determined increase in C4S in the malignant tissue. **(G)** Both the dominant negative SHP2 DNA construct and PHPS1 (30 μM x 24 h), a chemical SHP2 inhibitor, blocked DKK3 mRNA expression. In contrast, constitutively active SHP2 increased the mRNA DKK3 expression (p<0.001, n=6). These results indicate the involvement of SHP2 in the expression of DKK3. [ARSB=arylsulfatase B=N-acetylgalactosamine-4-sulfatase; CA=constitutively active; DKK=Dickkopf Wnt inhibitory factor; DN=dominant negative; DNMT=DNA methyltransferase; ERK=extracellular-signal regulated kinase; GALNS=galactosamine-(N-acetyl)-6-sulfatase; N-acetylgalactosamine-6-sulfatase; galactose-6-sulfate sulfatase; OE=overexpression; SHP2=non-receptor tyrosine phosphatase; si=siRNA].

Since inhibition of SHP2 increased the phospho-ERK1/2 in previous experiments [12], the impact of SHP2 inhibition was determined in the prostate stem cells. Dominant negative (DN) SHP2 markedly increased the phospho-ERK1/2, which was reduced by constitutively active (CA) SHP2 (p<0.001; n=3) (Figure 8C).

In the prostate stem cells, either ARSB knockdown or GALNS overexpression significantly inhibited the non-receptor tyrosine phosphatase SHP2 (PTPN11) activity (Figure 8D). Inversely, ARSB overexpression and GALNS knockdown significantly increased the SHP2 activity above the baseline level in the prostate stem cells (Figure 8D). The ARSB knockdown induced-decline in SHP2 activity was further reduced by the dominant negative (DN) SHP2 DNA construct (p<0.001, n=3), and the effect of ARSB silencing was inhibited by the constitutively active (CA) SHP2 DNA construct (p<0.001, n=3) (Figure 8E). In the malignant human prostate tissue, the SHP2 activity was reduced ∼50% (p<0.001, n=6; unpaired t-test, two-tailed) (Figure 8F).

The impact of changes in SHP2 on DKK3 expression was assessed in the prostate stem cells. Both the dominant negative SHP2 DNA construct and PHPS1, a chemical SHP2 inhibitor, blocked DKK3 mRNA expression. In contrast, constitutively active SHP2 increased the mRNA DKK3 expression (p<0.001, n=6). These results demonstrate a critical role for SHP2 in the regulation of DKK3 mRNA expression (Figure 8G).

### Pathway from phospho-ERK1/2 to inhibition of DKK3 expression involves nuclear-bound Myc/Max

Phospho-ERK1/2 impacts on the phosphorylation and activation of c-Myc [28, 29], and c-Myc interacts with DNMTs to affect DNA methylation [30, 31]. Hence, the impact of the chondroitin sulfatases and phospho-ERK1/2 on nuclear DNA-bound Myc/Max was addressed. Nuclear DNA-bound Myc/Max was significantly increased by ARSB silencing or GALNS overexpression (p<0.001, n=3). Inversely, ARSB overexpression and GALNS silencing reduced the Myc/Max binding (p<0.001, n=3) (Figure 9A). Treatment with the ERK activation inhibitor peptide I reversed the effect of GALNS OE on nuclear DNA-bound Myc/Max (Figure 9A). Nuclear DNA-bound Myc/Max was increased in the malignant prostate tissue, compared to the normal prostate tissue (p<0.001, unpaired t-test, two-tailed, n=6) (Figure 9B).

**Figure 9:** Impact of chondroitin sulfatases on DKK3 expression requires phospho-ERK1/2 and activation of c-Myc **(A)** Nuclear DNA-bound Myc/Max was detected by a transcription factor reporter assay (Signosis, Sunnyvale, CA) in nuclear extracts from control- and treated cell samples. A biotin-labeled c-Myc DNA binding sequence probe which detected Myc/Max bound to DNA was mixed with nuclear extracts to form c-Myc-DNA complexes. A filter plate was used to retain bound DNA probe and remove free probe, and the bound prelabeled DNA probe was eluted from the filter and collected for analysis. DNA-bound Myc/Max was significantly increased by both GALNS overexpression and ARSB silencing (p<0.001, n=3). Inversely, GALNS silencing and ARSB overexpression reduced the nuclear DNA-bound Myc/Max (p<0.001, n=3). The ERK activity inhibitor peptide I (10 μM x 24 h) effectively blocked the effect of GALNS overexpression, indicating a requirement for phospho-ERK1/2 for the GALNS overexpression-induced increase in nuclear DNA-binding of Myc/Max (p<0.001, n=3). **(B)** In malignant prostate tissue, the nuclear DNA-bound Myc/Max was ∼2.7 times the level in the normal tissue (p<0.001, n=6; unpaired t-test, two-tailed). **(C)** In the presence of a c-Myc inhibitor ((Z, E)-5-(4-Ethylbenzylidine)-2-thioxothiazolidin-4-one; 64 μM x 24 h) which inhibits Myc/Max dimerization, the increase in DNMT activity which followed ARSB silencing was inhibited (p<0.001, n=3). **(D)** Treatment by the c-Myc inhibitor increased the DKK3 mRNA following ARSB silencing (p<0.001, n=6), indicating a requirement for c-Myc in the ARSB knockdown-initiated inhibition of DKK3 expression. [ARSB=arylsulfatase B; DKK=Dickkopf Wnt inhibitory factor; DNMT=DNA methyltransferase; ERK=extracellular regulated kinase; GALNS=galactosamine-(N-acetyl)-6-sulfatase; N-acetylgalactosamine-6-sulfatase; galactose-6-sulfate sulfatase; Inh=inhibitor; OE=overexpression; si=siRNA].

When the prostate stem cells were treated with a c-Myc inhibitor, the increase in DNMT activity which followed ARSB-silencing was inhibited (p<0.001) (Figure 9C). The c-Myc inhibitor also blocked the ARSB-silencing induced decline in DKK3 expression (p<0.001) (Figure 9D).

### Schematic of the signaling cascade from chondroitin sulfatases to activation of Wnt/β-catenin signaling due to decline in DKK3

The schematic of the cascade initiated by changes in chondroitin sulfatases demonstrates a pathway from the inhibition of SHP2 by increased C4S. This pathway involves increases in phospho-ERK1/2, Myc/Max activation, and DNMT activity, leading to an epigenetic mechanism which can regulate Wnt signaling by increased methylation of the DKK3 promoter. Since DKK3 is an inhibitor of Wnt signaling, reduced DKK3 expression increases Wnt/β-catenin signaling (Figure 10).

**Figure 10:** Schematic of signaling pathway from chondroitin sulfates to the regulation of Wnt signaling by DKK (Dickkopf Wnt signaling pathway inhibitor)3 The signaling pathway from chondroitin sulfatases ARSB and GALNS involves changes in chondroitin 4-sulfation and chondroitin 6-sulfation, and leads to the inhibition of SHP2 activity due to increased binding with C4S. Decline in SHP2 activity leads to the sustained phosphorylation and activation of phospho-ERK1/2 and to the increased nuclear DNA binding of Myc/Max. DNMT activity and expression are also increased by changes in the chondroitin sulfatases, leading to increased promoter methylation of DKK3, reduced mRNA expression of DKK3, and increased activation of the Wnt pathway. The disinhibition of Wnt signaling due to reduced DKK3 expression leads to increased TCF/LEF nuclear DNA binding, increased nuclear β-catenin, and the increased expression of c-Myc and GATA-3. [ARSB=arylsulfatase B=N-acetylgalactosamine-4-sulfatase; C4S=chondroitin 4-sulfate; C6S=chondroitin 6-sulfate; DKK=Dickkopf; ERK=extracellular-signal regulated kinase; GALNS=galactosamine-(N-acetyl)-6-sulfatase; N-acetylgalactosamine-6-sulfatase; galactose-6-sulfate sulfatase; P=phosphate group; S=sulfate group; TCF-LEF=T-cell factor/lymphoid enhancer-binding factor].

## DISCUSSION

The experiments in this report show that the chondroitin sulfatases ARSB and GALNS contribute to the regulation of Wnt/β-catenin signaling by effects on the expression of Dickkopf Wnt signaling pathway inhibitor (DKK)3. By their effects on chondroitin sulfation, ARSB and GALNS regulate SHP2 activity. Decline in SHP2 activity causes sustained phosphorylation of substrates dependent on SHP2 phosphatase activity. This cascade of protracted phosphorylations, including increase in phospho-ERK1/2, can lead to profound changes in signaling, with effects on transcription, including hypermethylation of the DKK3 promoter and reduced DKK3 expression. Reduced DKK3 is anticipated to lead to increased Wnt/β-catenin signaling, possibly due to decline in inhibition of Wnt binding with its surface receptor complex, including low-density lipoprotein-related protein (LRP) 5/6 and Frizzled. Increased Wnt/β-catenin signaling is consistent with the study findings of increased nuclear β-catenin, nuclear DNA TCF/LEF binding, and mRNA expression of the Wnt-dependent genes c-Myc and GATA-3 following ARSB silencing or GALNS overexpression. The increased expression of c-Myc and GATA-3 was inhibited by blocking DNA methylation with 5-Azacytidine or by blocking β-catenin processing by JW67. In contrast, DKK3 mRNA expression was reduced by ARSB silencing and GALNS overexpression, and increased by 5-Azacytidine, indicating that a different underlying transcriptional mechanism was involved. In the experiments of this report, the inhibition of SHP2 activity by decline in ARSB or increase in GALNS leads to enhanced ERK phosphorylation, increased nuclear Myc/Max binding, increased expression and activation of DNA methyltransferases, and increased methylation of the DKK3 promoter. Reduced expression of DKK3 leads to disinhibition (increase) of Wnt signaling [9–11].

The mechanism by which the sulfatases affect DKK3 expression results from their impact on chondroitin 4-sulfation. Decline in ARSB leads to reduced degradation and increased accumulation of C4S. Increase in GALNS leads to decline in C6S and in chondroitin sulfate E (chondroitin-4,6-disulfate), leading to increases in the C4S to C6S ratio. SHP2 was previously shown to co-immunoprecipitate with C4S, leading to decline in SHP2 activity [12].

The crystal structure of SHP2 (PTPN11) was described almost 20 years ago [32]. The interactions of specific amino acids which determine the binding affinity of the phosphatase domain of SHP2 with phosphorylated tyrosine kinases has been well-described [13, 33, 34]. The auto-inhibition of SHP2, due to the presence of N-SH2 and C-SH2 domains and multiple tyrosine residues which can be phosphorylated, has been reported [13, 33–35]. The effect of the SHP2 inhibitor PHPS1 was attributed to the interaction of the sulfate (sulfonyl) group of PHPS1 with a specific binding site of SHP2 [13]. The SHP2/PHPS1-binding model indicated that the phenyl sulfonate group of PHPS1 acted as a phosphotyrosine mimetic, penetrating into the substrate-binding pocket of SHP2 [13]. We hypothesize that the sulfate group of N-acetylgalactosamine 4-sulfate, may also act as a phosphotyrosine mimetic and penetrate into the substrate binding pocket of SHP2. The amino acids at the periphery of the cleft where sulfate of PHPS1 binds are Lys-280, Asn 281, Arg-362, and His-426. These residues distinguish SHP2 from PTP1B, and may stabilize the anionic sulfate. Interaction of SHP2 with C4S may stabilize an inactive SHP2 conformation, or may bind SHP2 and prevent interaction with dephosphorylation targets, such as phosphorylated Ras [33–36].

The relationship between inhibition of SHP2 activity and malignancy is controversial, with some reports designating SHP2 as a proto-oncogene and suggesting that inhibition of SHP2 is advantageous in the treatment of malignancy [33, 34, 37–41]. In contrast, other investigations report that SHP2 activity is reduced in malignancy [12, 18, 42–45]. Decline in SHP2 has been associated with both activation and inhibition of cellular kinases [12, 18, 46–48]. Previous reports of proto-oncogenic effects of SHP2 and the benefits of SHP2 inhibition may be confounded by the use of vanadate [34, 49], since vanadate also inhibits sulfatase activity [50, 51]. Also, the time points in studies of effects of SHP2 on downstream signaling may be critically important, and may reflect fundamental differences in downstream signaling and activation in different cells and tissues. Also, studies that examine SHP2 expression, but not activity, may obscure the impact of SHP2 inhibition on downstream signaling.

The inverse effects between ARSB silencing or GALNS overexpression vs. ARSB overexpression or GALNS silencing present a novel and unanticipated reciprocity by which the C4S to C6S ratio is increased. The extracellular, endosulfatases Sulf1 and Sulf2, which remove 6-sulfate groups from N-acetylglucosamine-6-sulfate of heparan sulfate and heparin, have been reported to modify Wnt signaling [52, 53], but effects of GALNS or ARSB on Wnt signaling have not previously been reported. Future work will help to clarify how interventions to modify sulfatase activity impact on malignant transformation, differentiation, and proliferation. Differential binding of C4S or C6S with secreted molecules, including BMP4 and Wnt, may enable specific developmental responses. Small changes in ambient concentrations of oxygen, chloride, or other mediators, may lead to relative increase or decrease in sulfatase activity and, thereby, to changes in chondroitin sulfation [20, 54–56]. Previously, differences in expression of ARSB and GALNS between epithelium and stroma of developing rat prostate were reported [60]. The inverse effects of ARSB silencing and overexpression and GALNS overexpression and silencing suggest a well-demarcated separation of effects on Wnt/β-catenin signaling which may be highly relevant in developmental programming and malignant transformation.

## MATERIALS AND METHODS

### Cell culture and cell treatments

The human prostate stem cell line was obtained from ATCC (CRL-2887; Manassas, VA) and grown in Keratinocyte Serum Free Medium (K-SFM) with 0.05 mg/ml bovine pituitary extract (BPE) and 5 ng/ml epidermal growth factor (EGF), and maintained at 37°C in a humidified, 5% CO_2_ environment with replenishment of media every third day, as recommended. Confluent cells in T-25 flasks were harvested by EDTA-trypsin, and sub-cultured in multiwell tissue culture plates under similar conditions.

Cells were silenced for either ARSB (EC 3.1.6.12) or GALNS (EC 3.1.6.4) by specific siRNA (Qiagen, Germantown, MD) (see below). Overexpression of ARSB (NCBI NM_000046, transcript variant 1; TrueClone, OriGene, Rockville, MD) or of GALNS (NCBI NM_000512; TrueClone, Origene) was performed by transfection of specific untagged plasmids (see below), as previously [57]. Some cell preparations were treated with inhibitors added to the media for 24 h, including: PHPS1 (phenylhydrazonopyrazolone sulfonate, 30 μM; Sigma Chemical Company, St. Louis, MO), an inhibitor of SHP2; a cell-permeable inhibitor of ERK activation inhibitor peptide I (Ste-MPKKKPTPIQLNP-NH2, 10 μM; #328000, Calbiochem, San Diego, CA); c-Myc inhibitor, a cell-permeable thiazolidinone compound which inhibits c-Myc-Max dimerization (64 μM, 10058-F4, Tocris, Bio-Techne, Minneapolis, MN); JW67, an inhibitor of Wnt/β-catenin signaling by inducing β-catenin destruction (4 mg/ml, Tocris, Bio-Techne); and 5-azacytidine, an inhibitor of DNA methylation (10 μM, Sigma). Cells were harvested by scraping 24 h after silencing, overexpression, or treatment by chemical inhibitor.

### Human prostate tissue

Fresh frozen tissues from radical prostatectomies performed for prostate cancer were obtained from the University of Illinois at Chicago (UIC) Biorepository under a protocol approved by the Institutional Review Board and the Cancer Center of UIC. Frozen sections were performed and benign and malignant foci, consisting of epithelium and stroma, were identified, isolated, dissected out, and frozen for subsequent analysis, as previously [7, 8].

### Measurement of ARSB and GALNS activity

ARSB activity in the control and treated prostate stem cells and tissue was determined as reported previously [57]. Briefly, cells were harvested, and cell homogenates were prepared for measurement of ARSB activity. ARSB activity in the samples was determined using 4-methylumbelliferyl sulfate (MUS) as substrate in 0.05 M acetate buffer, pH 5.6. ARSB activity was determined using a standard curve of known concentrations of methylumbelliferyl, and was expressed as nmol/mg protein/h.

GALNS assay was performed with 5 μl cell homogenates made in ddH_2_O by sonication with a metal tip [57]. Homogenate was combined with 5 μl 0.2% heat-inactivated BSA (or 10 μl of 0.2% heat-inactivated BSA for blank) and 20 μl of substrate [10 mM 4-methylumbelliferyl-β-D-galactoside-6-sulfateNH_4_ (MU-βGal-6S)] in substrate buffer [0.1 M sodium acetate/0.1 M acetic acid at pH 4.3 with 0.1 M NaCl, 5 mM Pb-acetate (1.9 mg/ml) and 0.02% Na-azide] in wells of a microtiter plate. The plate was sealed, and incubated for 17 h at 37°C. Next, 5 μl 0.9 M Na-Phosphate buffer at pH 4.3 with 0.02% Na-azide was added, as well as 10 μl of 10 U β-d-Galactoside galactohydrolase (Sigma)/ml 0.2% heat-inactivated BSA. Reactants were incubated for 2 h at 37 °C, and then 200 μl of stop buffer [0.5 M NaHCO_3_/0.5 M Na_2_CO_3_ at pH 10.7 with 0.025% Triton-X-100] was added. Fluorescence readings were taken at 360 nm and 465 nm. GALNS activity was expressed as nmol/mg protein/h.

### ARSB and GALNS silencing by siRNA

Specific siRNAs for ARSB, GALNS and control siRNAs were procured (Qiagen) and used, as previously [57]. Briefly, cells were grown to 75% confluency in 12-well tissue culture clusters, and the medium of the growing cells was aspirated and replaced with 1.1 ml of fresh medium with serum. 0.3 μl of 20 μM siRNA (75 ng) was mixed with 100 μl of serum-free medium and 6 μl of HiPerfect Transfection Reagent (Qiagen). The mixture was incubated at room temperature for 10 minutes to allow the formation of transfection complexes, and then added dropwise onto the cells. The plate was swirled gently, and treated cells were incubated at 37°C in humidified 5% CO_2_ environment. After 24 h, the medium was exchanged with fresh growth medium. Efficacy of the silencing procedure was determined by measurement of ARSB and GALNS activity, as above.

### ARSB, GALNS and SHP-2 transfection

ARSB (NCBI NM_000046) and GALNS (NCBI NM_000512) plasmids in pCMV6-XL4 vector were obtained (Origene; http://www.origene.com/cDNA/default.mspx) and overexpressed in prostate stem cells by transient transfection using 2 μg of the plasmid and Lipofectamine™ 2000 (Invitrogen) [57]. Controls included untransfected cells and cells transfected with ARSB or GALNS vector control. Media were changed after 6 h, and cells were incubated in a humidified, 37°C, 5% CO_2_ environment and harvested 24 h after transfection. Similarly, SHP-2 dominant negative, constitutively active, wild type plasmid DNA, and empty vector were obtained (from Dr. Stuart Frank, University of Alabama at Birmingham) [58], and transfected in the prostate stem cells by Lipofectamine™ 2000. Efficiency of transfection was determined either by measuring ARSB or GALNS activity or by determination of SHP-2 protein by specific ELISA [18].

### Measurement of total sulfated glycosaminoglycans

Total sulfated glycosaminoglycan (GAG) content in cell lysates was measured using the sulfated GAG assay (Blyscan™, Biocolor Ltd., Newtownabbey, Northern Ireland), as previously [57]. The sulfated polysaccharide component of the proteoglycans (PGs) and the protein-free sulfated GAG chains were detected, whereas degraded disaccharide fragments or hyaluronan was not. The reaction was performed in the presence of excess unbound dye (1, 9-dimethylmethylene blue). Triplicate 50 μl samples (containing <5 μg of sulfated GAG and <250 mg cellular protein) were combined with 50 μl of deionized water in microcentrifuge tubes. Blyscan dye reagent (1.0 ml) was added, and tubes were mixed and shaken for 30 minutes. The cationic dye and GAG at acid pH produced an insoluble dye-GAG complex, forming a precipitate. The tubes were spun at 12,000 rpm for 10 minutes, and the unbound dye was removed. The Blyscan dissociation reagent (0.5 ml) was added and the bound dye was mixed into solution. The mixture was centrifuged at 12,000 rpm for 5 minutes. Then, 200 μl of each sample were transferred to wells of a 96-well plate and absorbance was read at 656 nm, the absorbance maximum of 1,9-dimethylmethylene blue, in a microplate reader (FLUOStar, BMG, Cary, NC). Readings were corrected by subtraction of the blank and compared to a standard curve prepared with known concentrations of sulfated GAGs. Concentration was expressed as micrograms/mg protein of cell or tissue lysate.

### Measurement of chondroitin 4-sulfate and chondroitin 6-sulfate

Chondroitin 4-sulfate monoclonal antibody (Clone LY111, AMS.A3143, Amsbio, Cambridge, MA) is specific for the native chondroitin 4-sulfate, not the chondroitin stubs. Cell lysates were prepared from treated and control cells. Chondroitin 4-sulfate was immunoprecipitated from the cell lysates, as previously [17, 57]. The precipitate was eluted with dye-free elution buffer and subjected to sulfated GAG assay, as above. Similarly, chondroitin 6-sulfate was immunoprecipitated from the cell lysates by a specific antibody (Clone MC21C, LS-C79286, LSBio, Seattle, WA) and processed further, as stated above.

### SHP-2 activity assay

SHP-2 Duo Set activity assay (R&D System, MN) was used to measure SHP-2 activity in control and treated prostate stem cells or in the prostate tissue homogenate of human normal and malignant prostate tissue. In this assay, an anti-SHP-2 antibody is conjugated to agarose immunoprecipitation (IP) beads and used to pull down both active and inactive SHP-2 in the samples. After washing away unbound material, a synthetic phosphopeptide substrate was added to the immunoprecipitates, and the substrate was dephosphorylated by active SHP-2 in the sample to generate free phosphate and unphosphorylated peptide. The beads were then pelleted by centrifugation, and the supernatant was transferred to a microplate. The amount of free phosphate in the supernatant was determined by a sensitive dye-binding assay using malachite green and molybdic acid. The activity of SHP-2 was determined from a phosphate standard curve.

### Nuclear DNA-bound Myc/Max assay

Activated Myc/Max binding to DNA was determined by a transcription factor reporter assay (Signosis, Sunnyvale, CA). Nuclear extracts were prepared from control and treated cell samples and from prostate tissue. Biotin-labeled, specific Myc/Max DNA binding sequence probe was mixed with nuclear extracts to allow formation of Myc/Max-DNA complexes. A filter plate was used to retain bound DNA probe and remove free probe. The bound pre-labeled DNA probe was then eluted from the filter and collected for quantitative analysis. The captured DNA probe was detected by streptavidin-HRP and specific luminescence substrate. Luminescence was measured as relative light units (RLUs) on a microplate luminometer (FLUOstar, BMG), and expressed as percentage of the untreated control preparation.

### Phospho-ERK1/2 ELISA

Cell extracts were prepared from both treated and control prostate stem cells in cell lysis buffer. Prostate tissue from normal and malignant human tissues were homogenized, and phospho-ERK1/2 [(Tyr(204/187)-Thr(202/185)] was measured in cell and tissue samples using a sandwich ELISA Kit (R&D Systems). A microtiter plate was coated with a capture antibody to total (phosphorylated and unphosphorylated) human ERK1/2. Samples and standards were added to the wells of the microtiter plate. Total-ERK1/2 in the lysates was captured by the coated antibody on the plate, and phospho-ERK1/2 was detected with biotinylated antibody to phospho-ERK1/2 and streptavidin-HRP. Hydrogen peroxide/tetramethylbenzidine substrate was used to develop the color which was proportional to bound HRP activity. The reaction was stopped, and the optical density of the color was read at 450 nm in a plate reader (FLUOstar). Phospho-ERK1, 2 concentrations in the sample were extrapolated from a standard curve obtained with known standards.

### DNA methyltransferase activity

DNA methyltransferase (DNMT) activity in nuclear extracts prepared from control and treated prostate stem cells and prostate tissues was determined by EpiQuik™ DNA Methyltransferase Activity/Inhibition Assay Kit (EpiGentek, Farmingdale, NY). In this assay, a unique cytosine-rich DNA substrate is stably coated on the test strip wells. DNMT enzymes in the samples transfer a methyl group to cytosine from Adomet (S-adenosylmethionine) to methylate the DNA substrate. The methylated DNA is recognized by an anti-5-methylcytosine antibody. The methylated DNA level was proportional to the enzyme activity, and was detected by a detection antibody, with enhancer and developer solutions. The developed color was quantified at 450 nm in a plate reader (FLUOstar).

### Methylation-specific PCR

Methylation-specific PCR was performed to detect the methylation status of the DKK3 gene promoter. Total DNA was isolated from cultured cells using the DNA Mini Kit (Qiagen). One μg of genomic DNA was bisulfate-treated with the EZ-DNA methylation Gold Kit (Zymo Research, Irvine, CA) and then resuspended in 10 μL Tris-EDTA buffer.

Two sets of DKK3 promoter primers were used to display the differences between methylated and unmethylated status. The primers targeting the unmethylated and methylated DKK3 promoter regions were:

DKK3 (Methylated) Forward: 5´-GGGGCGGGCGGCGGGGC-3´ and Reverse: 5´-ACATCTCCGCTCTACGCCCG-3´;

DKK3 (Unmethylated): Forward: 5´-TTAGGGGTGGGTGGTGGGGT-3´ and Reverse: 5´-CTACATCTCCACTCTACACCCA-3´.

The PCR products were visualized on a 2% agarose gel by ethidium bromide staining.

### Quantitation of DKK3 promoter methylation

DNA was isolated from the prostate stem cells and prostate tissue using the DNeasy Blood and Tissue kit (Qiagen). DNA was fragmented by sonication, and the MethylMiner™ Methylated DNA Enrichment Kit (ThermoFisher Scientific, Waltham, MA) was used for the enrichment and precipitation of methylated DNA. Precipitated, methylated DNA was further purified using the QIAquick PCR Purification kit (Qiagen). Methylated DNA was isolated from fragmented whole genomic DNA (5 ng - 25 μg) of the prostate stem cells and from the prostate tissue by binding to the methyl-CpG binding domain of human MBD2 protein, which was coupled to paramagnetic Dynabeads® M-280 Streptavidin using a biotin linker. The methylated fragments were then eluted as a single enriched population with 2000 mM NaCl elution buffer. The eluted methylated dsDNA was then subjected to real-time PCR assays with specific primers to the DKK3 promoter. Promoter primers were: (forward)-5´CATCACAGGTGAGGAGCAGA-3´ and (reverse): 5´-AAACGCAGCTCCCCTACAC-3´. The methylated DNA was quantified using standard analysis methods for QPCR [57].

### QRT-PCR for DNMT 1, 3a, 3b, DKK3, c-Myc, GATA3, ARSB, and GALNS

Total RNA was prepared from control and treated cells using an RNeasy Mini Kit (Qiagen), and QRT-PCR was performed using specific primers and previously described quantitative methods [57]. Primers were selected for DNMT1, DNMT 3a, DNMT 3b, ARSB, GALNS, DKK3, c-Myc, and GATA3. The primers were:

DNMT 1 (NM_001130823.2) Forward: 5´-CCTAGCCCCAGGATTACAA-3´ and Reverse: 5´-ACTCATCCGATTTGGCTCT-3´;

DNMT 3a (NM_001320893.1) Forward: 5´-CCGATGCTGGGGACAAGA-3´ and Reverse: 5´-CCCGTCATCCACCAAGAC-3´; and

DNMT 3b (NM_001207055.1) Forward: 5´-CCCAGCTCTTACCTTACCA-3´ and Reverse: 5´-GGTCCCCTATTCCAAACTC-3´.

ARSB (NM_000046) Forward: 5´-AGACTTTGGCAGGGGGTAAT-3´ and Reverse: 5´-CAGCCAGTCAGAGATGTGGA-3´;

GALNS (NM_000512) Forward: 5´-ACGGATTTGATG AGTGGTTTG-3´ and Reverse: 5´-GTAGAGGAAAAAGGGGTGGTG-3´.

GATA-3 (X55037): Forward: 5’-AGACCACCACAACCACACTCT-3’ Reverse: 5´ – GCCTTCCTTCTTCATAGTCAGG-3’

c-Myc (NM_00246.7) Forward: 5’-GGAGGCTATTCTGCCCATTT-3’ Reverse: 5’-AGGCTGCTGGTTTTCCACTAC-3’.

DKK3 (NM_015881.5) Forward: 5´-CGAGGTTGAGGAACTGATGG-3’ Reverse: 5´-CCTTCGTGTCTGTGTTGGTCT-3’.

### Nuclear β-catenin assay

Nuclear β-catenin was measured in control and treated cell samples and prostate tissues using a sandwich ELISA (R&D Systems, Minneapolis, MN), as previously [59]. Nuclear extracts were prepared, and a sandwich ELISA was used to capture the β-catenin. The optical density of the color was read at 450 nm in a plate reader (FLUOstar). The nuclear β-catenin concentrations in the samples were extrapolated from a standard curve derived using known standards.

### TCF/LEF (T-cell factor/lymphoid enhancer-binding factor) assay

Binding of TCF/LEF to DNA was determined by a transcription factor reporter assay (Signosis, Sunnyvale, CA). Nuclear extracts were prepared from control and treated prostate stem cells. TCF/LEF binding to a specific DNA sequence was determined by a specific Biotin-labeled TCF/LEF DNA probe. The captured DNA probe was detected by streptavidin-HRP and specific luminescence substrate. Luminescence was measured and expressed as a percentage of the untreated control.

### Statistical methods

Data presented are the mean ± SD of at least three independent experiments. Mean values for each sample were calculated as the average of two technical duplicates of each measurement. Data presented in the text and figures are representative of multiple independent experiments. Statistical significance was determined by one-way analysis of variance followed by post-hoc Tukey’s test for multiple determinations using InStat3 software (GraphPad, La Jolla, CA), unless stated otherwise. Unpaired t-tests, two-tailed, were used for two-way comparisons. P values ≤ 0.05 are considered to be statistically significant and are indicated by ^*^. ^**^ represents p< 0.01, ^***^ for p< 0.001 and ^****^ for p< 0.0001. # signs are used to indicate declines from baseline control levels, and ### represents p<0.001.
